# Analysis of Older Adults under Home Care in Taiwan's Ageing Society

**DOI:** 10.1155/2022/8687947

**Published:** 2022-06-21

**Authors:** Jhih-Ling Chiu

**Affiliations:** Department of Risk Management and Insurance, Ming Chuan University, Taipei, Taiwan

## Abstract

As of January 2022, 16.91% of Taiwan's population was over the age of 65, and a 2017 study indicated that 94.2% of patients who required long-term care in Taiwan received home care. This study produced a “post-home care patient information survey” to understand the characteristics of home care patients and the volume and results of home care and investigate the relationships between them. Different diagnoses were found to have no significant effect on the volume or results of home care. Positive correlations were found between the services patients required and the volume of home care and specific results. Volume and specific results were also positively correlated. The termination of home care was primarily due to medical needs (98.6%). As the Taiwanese population ages, home care must be improved, and the conditions for which patients can receive home care should be expanded. Care services should replace diagnoses in determining benefit standards for home care payments.

## 1. Introduction

As of January 2022, people over 65 accounted for 16.91% of Taiwan's total population, making Taiwan an aged society [1]. The World Health Organization and United Nations definition of an aged society is one in which no less than 14% of the population is over the age of 65.2. Furthermore, Taiwan is expected to be classified as a superaged society by 2026, at which point, more than 20% of the population will be over the age of 65 [2, 3].

As the Taiwanese population continues to age and overall life expectancy rises, this has led to increases in functional impairments, disability, and the incidence of chronic diseases [4]. Concomitantly, the demand for long-term care in Taiwan has risen. In 2017, only 5.8% of all long-term care patients used institutional care, while 94.2% received home-based care [5]. Home care patients often have multiple comorbidities, which is demonstrated by the fact that 90.04% are classified into resource utilization groups 2 and 3 [6, 7]. These patients require one or two additional specialized care services over and above ordinary healthcare services provided to group 1-classified patients. Together with the socioeconomic diversity of patients, these requirements place further demands and stresses on home healthcare [7].

Home care can be defined as health care services provided to a patient in a familiar environment, where families can care for patients with modern medical measures and professional assistance without general hospital facilities and services [8]. Current home care services in Taiwan include housework and daily care (washing and mending clothing, correspondence, food preparation, etc.) and physical care (bathing, taking medication, rolling over, etc.). Home care has several advantages, including assisting in managing healthcare facility capacity constraints, reducing the risk of nosocomial infections, and improving continuity of care while lowering readmission and mortality risks [4].

The predictors of the types and duration of home care services remain contested in the literature, with patient diagnosis, mobility during care, and nursing problems being argued as being more critical [9, 10]. The duration of home care has been demonstrated to increase as patients' ability to care for themselves diminishes [11]. In addition, patients' diagnoses, nursing problems, and required care accurately predicted the cost of care and mobility at the end of care [12]. The evaluation of home care can be separated into overall and specific outcomes [13]. Overall outcomes refer to the improvement or stability of patients' ability to function in daily life and their levels of dependence and consciousness. In contrast, specific outcomes refer to the number of comorbidities and hospital stays during care.

This study aimed to investigate the characteristics of home care patients, the volume of home care, and the outcomes of care that could be used to help identify home care needs, assist caregivers in organizing adequate care for older adults, and determine how these characteristics may impact the volume of home care and their outcomes.

## 2. Materials and Methods

This study was structured based on literature review and practical experience. Surveys were used to assess the volume of home care (number of home visits and phone calls by nurses and number of home visits by doctors during home care) and the outcomes of home care (overall outcomes: changes in mobility and consciousness during and after care; specific outcomes: number of hospital visits, number and duration of hospital stays, and comorbidities during home care). Analysis was performed on home care patient information and logs from January to March of 2014 at 38 registered home care institutions in Taiwan. The conditions and evaluation tools for home care in a long-term care system and the actual investigation of patient information were used to draft a “post-home care patient information survey” as detailed below:

1. Basic patient information: gender, age, marital status, place of residence, cohabiting family members, main caregiver, household income, origin of home care referral, reason for terminating home care, and reason for terminating care.
2. Patient illness information: diagnosis and care services at start of home care.
3. Patient home care information: volume of home care (number of home visits and phone calls by nurses and number of home visits by doctors during care) and home care outcomes (specific and overall).

The completed “home care patient information survey” was edited after discussing its appropriateness with two nurses from a medical center. Afterward, it was sent to three home care nursing professionals to review content validity. These professionals examined and edited the accuracy, applicability, and inclusiveness of the content. The investigator conducted a pilot study at two home care facilities affiliated with a single medical center where the investigator and two nurses each recorded the information for ten patients to assess consistency across those who recorded the information. The investigator conducted a pilot study at two home care facilities where the information for ten patients was recorded to assess consistency. Surveyor reliability was 0.88 (*r* = 0.88). The reliability of the survey itself was retested; information for another ten patients was recorded and then rerecorded one week later. The new reliability was 0.97 (*r* = 0.97). The validity and reliability tests for this survey were used to understand the characteristics and care information of home care patients.

The investigator requested home care professionals at an April 2012 cross-strait medical conference to record information for their January–March 2014 postcare patients. Information was collected for a total of 427 postcare patients. After processing the collected data, average, mean, analysis of variance, and chi-squared test statistical analyses were conducted using the SPSS/PC + software.

Ethical approval for this study and written informed consent from the participants of the study were not required in accordance with local legislation, and national guidelines as no human or animal studies are presented in the manuscript.

## 3. Results

Table 1 shows basic personal information for the 427 postcare patients.  Table 2 shows the types of home care services required by patients under different diagnosis classifications. 156 patients (36.5%) required a total of 1–5 care services; 216 patients (50.6%) required 6–10 care services; 55 patients (12.9%) required 11 or more care services. For volume of home care, the average duration of care was 215.08 days (SD = 310.88); the average number of nurse visits was 13.41 (SD = 17.89); the average number of nurse phone calls was 10.58 (SD = 16.10); the average number of doctor visits was 1.47 (SD = 3.99).  Table 3 details the specific outcomes for postcare patients.  Table 4 shows the overall outcomes for postcare patients.

Analysis of variance found that diagnosis classifications had no significant effect on home care information (*p* > 0.05). There were no significant differences in the volumes or specific outcomes of home care for patients with different diagnosis classifications. Chi-squared tests found no correlation between diagnosis and overall outcomes (mobility and consciousness).  Table 5 shows a positive correlation between the number of services required and the volume and specific outcomes (*p* < 0.001); however, after dividing the amount of care needed into 1–5, 6–10, and greater than 10 services, chi-squared tests found no correlation between the number of services and overall outcomes. Chi-squared tests showed no correlation between the volume of home care (turned into category variables) and overall outcomes of home care, and a positive relationship between the volume of home care and specific outcomes of home care (*p* < 0.001).

## 4. Discussion

When home care specialists visit patients, they do more than simply administer care; they teach and provide an example for patients and their families on how to take care of themselves [14]. Patients who require more services most likely have more severe illnesses and a higher volume of needed care. Comorbidities (especially pressure sores) for patients also clearly increase while receiving home care, which is a significant challenge for home care specialists as increased comorbidities further add to the duration and volume of care required. Patients receiving home care all have some form of chronic illness. The goal of their home care is mainly to manage symptoms and prevent further deterioration of health, and the presence of comorbidities can hasten the progression of their disease. Given that 98.6% of patients terminated home care due to medical needs, it is clear that the current state of home care in Taiwan is not adequate.

The structured survey in this study provided insight into the long-term care of home care patients. The significant findings are summarized below:

1. 76.1% of those receiving home care are older adults; 97.4% of patients live with their families; 98.6% of patients terminated home care due to medical needs.
2. The average duration of care for postcare patients was 215.08 days; the average number of nurse home visits was 13.41; the average number of nurse phone calls was 10.58; the average number of doctor home visits was 1.47; the average number of visits to a clinic was 1.93; the average number of hospital stays was 0.42; the average length of hospital stays was 4.99 days.
3. Different diagnosis classifications had no significant effect on the volume or outcomes of home care. However, the types of services patients required were positively correlated to the volume of home care and the specific outcomes.
4. The volume of home care and specific outcomes were positively correlated. Different diagnosis classifications were found to have no significant effect on the volume or outcomes of home care. The types of services patients required were positively correlated to the volume of home care and the specific outcomes. The volume of home care and specific outcomes were positively correlated.

As patients mainly require emotional consultation and advice, home care specialists are advised to strengthen communication skills. It is also essential for nurses to attend home care specialist training to acquire the wide range of skills required for home care patients.

As Taiwan's society continues to age, home care must be improved, and its requirements should be broadened to include patients with mild dependence (levels 0–1) that require medical treatment and care. Care services should also replace diagnoses in determining benefit standards for home care payments. Future standardization of home care institution logs can also increase data accuracy and reliability.

## 5. Additional Points

There were several limitations to this study worth noting:

1. The duration of care for postcare patients was difficult to determine as some home care institutions did not consider short hospital stays as having closed cases.
2. Despite the advances in information technology, there is a significant disparity between the logs kept at different institutions. The disparity created difficulty when comparing raw data from each home care institution.
3. Many institutions were unwilling to provide certain information, especially involving income, possibly due to competition.

Patient information logs must be standardized for future research to thoroughly compare home care institutions. Standardized data collection forms can increase the accuracy and reliability of the data collected. Once records are standardized, collecting national home care data, or comparing different locations and institutions will become more effective. The gathered long-term care patient information could then more clearly quantify postcare outcomes and serve as a reference for long-term care insurance institutions when establishing standards for home care service fees.

## Figures and Tables

**Table 1:** Basic personal information.

Item	No. of persons	%
*Gender*		
Male	211	49.4
Female	216	50.6

*Place of residence*		
Urban area	221	51.8
Rural area	206	48.2

*Marital status*		
Married	273	63.9
Single	154	36.1

*Cohabiting family members*		
Lives alone	11	2.6
Lives with others (spouse, children)	416	97.4

*Main caregiver*		
Spouse	114	26.7
Family or friends (other than spouse)	225	59.7
Private worker	58	13.6

*Household income*		
Upper class	113	26.5
Middle class	266	62.3
Lower class	48	11.2

*Reason for terminating home care*		
Medical needs	421	98.6
Family burden	6	1.4

*Reason for terminating care*		
Illness improved	68	15.9
Illness worsened	89	20.9
Family reasons	50	11.7
Death	220	51.5

**Table 2:** Types of home care services required for patients with different diagnosis classifications.

Care service	Category 1		Category 2		Category 3	
	*n* = 47		*n* = 285		*n* = 95	
	No. of persons	%	No. of persons	%	No. of persons	%
General physical examinations	45	95.7	246	86.3	79	83.2
Monitoring of vital signs	46	97.9	261	91.6	87	91.6
Nursing instruction (nutrition, medication)	45	95.7	262	91.9	86	90.5
Injections (I.M., S.C., I.V.)	2	4.3	16	5.6	18	18.9
Adding medication to IV bags (chemotherapy, pain management)	0	0.0	5	1.8	17	17.9
Passive joint movement	25	53.2	178	62.5	38	40.0
Changing catheters and catheter bags	24	51.1	125	43.9	45	47.4
Oral care	11	23.4	98	34.4	31	32.6
Suppository administration	3	6.4	19	6.7	1	1.1
Sending test samples	10	21.3	62	21.8	25	26.3
Drawing blood for tests (blood sugar, etc.)	12	25.5	85	29.8	31	32.6
IV bags (blood transfusions)	0	0.0	10	3.5	15	15.8
Testing for drug reactions	0	0.0	2	0.7	3	3.2
Bathing	3	6.4	17	6.0	8	8.4
Washing hair	0	0.0	3	1.1	1	1.1
Catheterization	5	10.6	25	8.8	7	7.4
Enema	0	0.0	11	3.9	4	4.2
Inserting or changing nasogastric tubes	21	44.7	203	71.2	38	40.0
Respiratory tract suction (removal of sputum)	5	10.6	62	21.8	21	22.1
Postural drainage	4	8.5	27	9.5	5	5.3
Changing medication	14	29.8	106	37.2	32	33.7
Removal of faecal impaction	2	4.3	14	4.9	7	7.4
Lavage of anus praeter naturalis	1	2.1	1	0.4	1	1.1
Cystostomy and gastrostomy care	1	2.1	5	1.8	4	4.2
Bladder irrigation	3	6.4	13	4.6	6	6.3
Perineum washing	4	8.5	28	9.8	6	6.3
Changing tracheotomy tube	4	8.5	48	16.8	17	17.9
Tracheotomy incision	4	8.5	37	13.0	12	12.6
Steam inhalation therapy	1	2.1	15	5.3	4	4.2
Equipment rental	3	6.4	6	2.1	3	3.2
Other	0	0.0	3	1.1	6	6.3

**Table 3:** Specific outcomes of home care patients.

			Average		Standard deviation	
Number of clinic visits			1.93		7.36	
Number of hospital stays			0.42		0.83	
Length of hospital stay (days)			4.99		12.05	

No. of comorbidities			No. of persons		%	
0			154		36.1	
1–2			208		48.7	
3–4			57		13.3	

Comorbidity	Category 1		Category 2		Category 3	
	*n* = 47		*n* = 285		*n* = 95	
	No. of persons	%	No. of persons	%	No. of persons	%

No comorbidities	18	38.30	98	34.4	38	40.0
Pressure sores	17	36.2	91	31.9	23	24.2
Upper respiratory tract infection	5	10.6	69	24.2	9	9.5
Falls	1	2.1	3	1.1	4	4.2
Burns	0	0.0	1	0.4	1	1.1
Pneumonia	1	2.1	28	9.8	7	7.4
Fractures	0	0.0	1	0.4	1	1.1
Urinary tract infection	17	36.2	50	17.5	20	21.1
Gastrointestinal bleeding	0	0.0	22	7.7	0	0.0
Faecaloma obstruction	4	8.5	50	17.5	20	21.1
Contracture	3	6.4	8	2.8	7	7.4
Other (dermatosis, oedema, low blood sugar)	6	12.8	22	7.7	3	3.2

**Table 4:** Overall outcomes of home care patients.

Item	No. of persons	%
*Mobility during care (Karnofsky scale)*		
Level 0	2	0.5
Level 1	2	0.5
Level 2	16	3.7
Level 3	89	20.8
Level 4	318	74.5

*Mobility after care (Karnofsky scale)*		
Level 0	2	0.5
Level 1	5	1.2
Level 2	22	5.2
Level 3	68	15.9
Level 4	330	77.3

*Changes in mobility during and after care*		
Improved	27	6.3
No change	374	87.6
Worsened	26	6.1

*Consciousness during care*		
Conscious	96	22.5
Confused	196	45.9
Comatose	135	31.6

*Consciousness after care*		
Conscious	85	19.9
Confused	114	26.7
Comatose	228	53.4

*Changes in consciousness during and after care*		
Improved	23	5.4
No change	297	69.6
Worsened	107	25.1

Karnofsky scale: level 0: full mobility; level 1: able to walk and do mild work; level 2: able to take care of themselves; unable to do office work; most time is spent out of bed or wheelchair; level 3: can only take limited care of themselves; most time is spent in bed or wheelchair; level 4: not mobile.

**Table 5:** Relationship between specific outcomes, care, and volume of home care (*n* = 427).

Correlation value			Volume of care		
Length of care			0.34^*∗∗*^		
Number of home visits			0.38^*∗∗*^		
Number of phone calls			0.34^*∗∗*^		
Number of doctor visits			0.21^*∗∗*^		
Number of clinic visits			0.20^*∗∗*^		
Number of hospital stays			0.22^*∗∗*^		
Length of hospital stay (days)			0.17^*∗∗*^		
Comorbidities			0.49^*∗∗*^		

Correlation value	Comorbidities	Number of clinic visits		Number of hospital stays	Length of hospital stay (days)

Volume of care	0.39^*∗∗*^	0.28^*∗∗*^		0.41^*∗∗*^	0.28^*∗∗*^
Number of home visits	0.46^*∗∗*^	0.37^*∗∗*^		0.44^*∗∗*^	0.27^*∗∗*^
Number of phone calls	0.30^*∗∗*^	0.29^*∗∗*^		0.34^*∗∗*^	0.21^*∗∗*^
Number of doctor visits	0.19^*∗∗*^	0.14^*∗∗*^		0.24^*∗∗*^	0.14^*∗*^

*∗*, *p* < 0.01; ^*∗∗*^, *p* < 0.001.

## Data Availability

The data that support the findings of this study are available from the corresponding author upon reasonable request.
